The article "Analysis and Research on Sustainable Development Factors of the Sports Industry Based on Chaos Theory" was published in 2022. Journal: J Environ Public Health.

# Analysis and Research on Sustainable Development Factors of the Sports Industry Based on Chaos Theory

**DOI:** 10.1155/2022/1060639

**Published:** 2022-06-14

**Authors:** Yuankai Luo, Shanshan Gao, Xuanfei Yan, Yecheng Cao

**Affiliations:** ^1^Department of Physical Education, Guangdong Technology College, Zhaoqing 526100, China; ^2^Department of Physical Education, Shijiazhuang University, Shijiazhuang 050035, China

## Abstract

The sports industry is an emerging industry with broad development prospects, and it is also full of competition. The sports industry has the characteristics of fluctuation, intermittence, and randomness, which are suitable for the analysis of chaos theory in order to find out the internal development law of the sports industry. In order to solve the above problems, an improved chaos theory method is proposed in this paper and the *K*-cluster analysis method is integrated into chaos calculation, in order to reduce the occurrence rate of the “local extreme value” and improve the accuracy of calculation results. The model uses nonlinear and irregular chaos theory to analyze the aggregation degree of sports industry, industrial spatial distribution, and the spatial governance effect and find out the best optimization decision. When selecting the optimization indicators, not only the European distance of each indicator cluster but also the spatial correlation of the indicators are considered to realize the comprehensive analysis of the sports industry and improve the accuracy of optimization. In the simulation analysis of optimization decision-making, the decision-making model based on chaos theory is compared with the previous first-order decision-making model. The results show that the improved chaos theory can control the data aggregation range of sports industry between (0∼3), the data fusion degree of industrial space between 95 and 99%, and the variation range between 0 and 0.2%, which is significantly better than (0∼9), 90∼95%, and 0∼0.4% of the genetic algorithm. Therefore, the aggregation degree, spatial governance, and decision optimization of the optimization decision-making model proposed in this paper are better than those of the previous genetic algorithm.

## 1. Introduction

Chaos theory is a method with both qualitative thinking and quantitative analysis. It is used to explore the behavior in dynamic systems (such as population movement, chemical reaction, meteorological change, and social behavior) that can only be explained and predicted with a whole continuous rather than a single data relationship.

Chaos is not an accidental or individual event but a universal phenomenon in all kinds of macrosystems and microsystems in the universe. Everything is chaotic. Chaos is not an independent science either. It promotes and depends on each other with other sciences, which leads to many interdisciplinary subjects, such as chaotic meteorology, chaotic economics, and chaotic mathematics. Chaos is not only of a great research value but also of a practical application value. It can directly or indirectly create wealth. Theoretically, the purpose of studying chaos is multifaceted: revealing the essence of chaos (internal randomness), describing its basic characteristics, understanding its dynamic behavior, and striving to control it for the human use. In the past 20 years, chaos has gradually changed from a harmful phenomenon to a phenomenon with a practical application value in engineering systems. A lot of research work in recent years shows that chaos is more and more closely related to engineering technology. It has a wide range of applications in biomedical engineering, kinetic engineering, chemical reaction engineering, electronic information engineering, computer engineering, applied mathematics, and experimental physics. In the aspect of application, it mainly includes chaotic signal synchronization and secure communication, chaotic prediction, information processing of the chaotic neural network, chaotic and fractal image processing, optimization method based on chaos, chaotic bioengineering, weather system, ecosystem, and chaotic economy. In addition, the technology of controlling chaos has also been applied to the research of neural networks, lasers, chemical reaction processes, hydrodynamics, nonlinear mechanical fault diagnosis systems, nonlinear circuits, celestial mechanics, medical treatment, and physical systems with distributed parameters. At present, in some fields where chaos is very important and useful, purposeful generation or enhancement of chaos has become a key research topic. Chaos theory has been applied in educational administration, curriculum and teaching, educational research, educational testing, and so on. Because the object of education is people, people are individuals who change and fluctuate at any time and the process of education basically follows certain guidelines and has experienced long-term interaction, which is quite in line with the framework of chaos theory. Therefore, according to the chaos theory, the education system is easy to produce unexpected results. This result may be positive or negative. Whether positive or negative, what is important is that, in addition to short-term observations, long-term data should be accumulated to analyze the possible context so as to increase the predictability of the educational effect and use it to expand the educational effect.

The article "Analysis and Research on Sustainable Development Factors of the Sports Industry Based on Chaos Theory" was published in 2022. Journal: J Environ Public Health.

In view of the social concern for public health and the harm brought by unscientific sports, countries all over the world are sparing no effort to develop sports. Ahmad and Shin proposed that the sports industry is the fastest growing and most mature sports industry [1], which has the basic conditions and policy conditions for large-scale development. According to the latest statistics of the WHO in 2020, the number of participants in China's sports industry will reach 452.01 million in 2022. However, the level of participation in public health is about 56.3% of the global average, indicating that the development of China's sports industry lags behind. Altinay and Kozak proposed there were many nonlinear algorithms, mainly including time series, Kalman filter, adaptive fuzzy logic, artificial neural network, grey prediction, wavelet analysis, and chaos theory algorithms [2]. Ataei et al. proposed among them, the chaos theory algorithm was first used to analyze atmospheric convection and then gradually applied to sports-related industries [3]. Chen and Yang proposed through dimensionality reduction analysis that the theoretical algorithm makes a “short analysis” of “continuous data,” which can analyze massive sports data, standardize the nonlinear and irregular fitness needs, calculate the aggregation degree and spatial distribution standard of the sports industry, and provide support for the spatial governance decision-making of the sports industry [4]. Drezet proposed that the results show that the chaos theory model is closer to the actual public demand in terms of sports industry agglomeration and sports spatial distribution [5]. Gonzalez-Serrano et al. proposed the advantages of strong discrete data processing and reasonable spatial distribution design, which can meet the actual needs of public health [6]. Kania also put forward the model algorithm of chaos theory and spatial optimization [7]. Li et al. proposed that the results show that the chaotic model was significantly better than the previous qualitative analysis methods in terms of data processing capacity and data processing efficiency, such as artificial neural network, and grey prediction [8]. At the same time, the algorithm provides clear guidance and opinions for the development, structural optimization and spatial rational distribution of the local sports industry and finds out the potential points of the development of the sports industry. Miandoab had shown that there was a close relationship between the degree of sports industry agglomeration and spatial governance [9].

Peng et al. proposed that we need to integrate the characteristics of the two before we can play the iterative role of 1 + 1 > 2 [10]. Vergini proposed the key to the development and improvement of the sports industry was to deeply analyze the guidance of chaos theory on sports industry agglomeration and spatial governance and build an industrial agglomeration and the spatial governance model based on chaos theory [11]. According to the above research status, the common method of sports industry agglomeration is chaos theory and the genetic algorithm, scholars generally believe that chaos theory cannot deal with large-scale sports industry data and there is a problem of a high “local extreme value” rate, resulting in deviation in the calculation results. Some scholars also proposed that the *k*-clustering method can reduce the occurrence rate of “local extremum.” Therefore, based on the previously mentioned research, this paper creatively improves the chaos theory and method, integrates the *k*-clustering method, and constructs the improved models of industrial agglomeration, sports industrial agglomeration, and spatial governance. In order to verify the accuracy of the model, it is compared with the genetic algorithm commonly used in the sports industry. It is mainly divided into three parts: the first part expounds the research status of sports industrial agglomeration and spatial governance; the second part constructs the sports industry agglomeration and the spatial governance algorithm based on the chaos theory and explains the self-learning, extreme value judgment, and conditional constraints in the model; the third part verifies and analyzes the concentration and spatial governance of the sports industry based on mixed theory and draws the research conclusion of this paper. Compared with other literature studies, the innovation of this paper is to propose a chaotic theoretical model for sports industry agglomeration and spatial governance, analyze the irregularity of discrete data in the sports industry, and put forward targeted optimization decisions. Firstly, self-learning and constraints can identify the characteristic data in the sports industry and the similarity between aggregation and spatial governance. Secondly, extreme value judgment can improve the accuracy of sports industry agglomeration and spatial governance.

The article "Analysis and Research on Sustainable Development Factors of the Sports Industry Based on Chaos Theory" was published in 2022. Journal: J Environ Public Health.

## 2. Description of Sports Industry Agglomeration and Spatial Governance Based on Chaos Theory

Firstly, using the irregular and nonqualitative analysis logic in the chaos theory, this paper identifies the four parameters of the sports industry agglomeration and spatial governance (intraindustry agglomeration, interindustry agglomeration, regional spatial governance, and overall spatial distribution governance). Secondly, governance decision-making is built and the optimization goal of the sports industry is achieved. The optimization index system of industrial agglomeration and spatial governance determines each judgment index and index content. Finally, using the delay factors (time factor, regional factor, and event factor) in chaos theory, the trajectory of the obtained sports industry data is analyzed; finally, the conclusion of nonlinear and irregular chaos is drawn. The specific data processing process is shown in Figure 1.

Through the sports industry data released by local governments, 1200 survey documents and 56 interview information, 55 indicators of sports industry agglomeration and spatial governance are obtained and the validity and reliability of each indicator are >0.7. Among them, the data released by the government are the 10-year data from 2011 to 2021 and the questionnaire is the result obtained in 2021. In June of the same year, 56 experts were interviewed from 6 provinces in the southeast, 4 provinces in the northeast, and 2 provinces in the northwest. The weight of the obtained indicators is calculated and analyzed, and the weight range is 0∼1, which is closer to 1. It can be seen that the indicators obtained from the questionnaire are good, as shown in Table 1.

## 3. Analysis of the Optimization Decision Model of Sports Industry Agglomeration and Spatial Governance Based on Chaos Theory

### 3.1. Sports Industry Agglomeration Based on Chaos Theory

In the development of the sports industry, the rightmost effect of industrial agglomeration is found through the identification of the degree of agglomeration. Chaos theory analyzes the aggregation within and among industries, judges the development level and the degree of different sports in the sports industry, and formulates the development plan of the sports industry according to the actual aggregation situation. In the process of analyzing the degree of agglomeration, Wang et al. proposed that we should pay attention to the correlation between the sports industry and derivative industries, as well as the correlation within and among industries, and the necessary weights should be set to obtain the degree of industrial agglomeration more accurately [12]. Wang proposed that due to the limitations of sports habits, local customs, and seasons, there are often high deviations in the aggregation results of the sports industry [13]. In order to reduce the above deviation and reduce the influence of factors on the results, it is necessary to restrict and differentiate the sports industry and eliminate the influence of irrelevant factors. In addition, the aggregation degree of the sports industry should be constrained, and the final aggregation result should be obtained through iterative calculation. The aggregation process of the sports industry is shown in Figure 2.

The article "Analysis and Research on Sustainable Development Factors of the Sports Industry Based on Chaos Theory" was published in 2022. Journal: J Environ Public Health.

In the process of sports industry agglomeration analysis, customs, seasons, and regions affect the whole sports industry and have a consistent impact on the agglomeration of the sports industry. Therefore, chaos theory should deal with the information in the sports industry agglomeration irregularly, realize the discontinuous analysis of the sports industry, and reduce the impact of the above factors on the sports industry agglomeration.

### 3.2. Spatial Governance of the Sports Industry Based on Chaos Theory

Xu and Yang proposed that the development of the sports industry changes with space and presents different spatial characteristics through the nonlinear influence of different infrastructure [14]. When the constraints are fixed, the steps of spatial governance will be simplified, but the governance result was still not a constant value because of the changes of the spatial governance of the sports industry. Therefore, the spatial governance of the sports industry presents dynamic changes. Chaos theory regards the spatial governance of the sports industry as a time series, and then, the time series contains not only the external data of the spatial governance of the sports industry but also the internal data of the spatial governance of the sports industry. Therefore, to improve the accuracy of spatial governance of the sports industry is to construct a chaotic time series. The specific sequence results are shown in Figure 3.

It can be seen from Figure 3 that different governance schemes are adopted for different sports industry contents. At the same time, the irregular computing concept of the chaos theory can be spatially controlled through orderly time. According to the difficulty of space governance of different sports events, long-term, and short-term governance schemes are adopted to achieve the optimization purpose of space governance.

### 3.3. Construction of the Spatial Governance Algorithm of the Sports Industry Agglomeration Area Based on Chaos Theory

Suppose that the sports industry aggregation is *x*_*i*_ represents the cohesion of the sports industry, and *j* represents the aggregation among the sports industries; then, *x*_*ij*_ represents the aggregation of any item in the sports industry. The spatial governance of the sports industry is *y*_*i*_ that represents regional spatial governance, *j* represents overall spatial governance, and *y*_*ij*_ represents the spatial governance of any project in the sports industry. Suppose that the sports industry items are *N* = {*n*_1_*,n*_2_,…*,n*_*i*_}, *n*_*i*_=∑_*i*,*j*_^*∞*^*f*(*x*_*ij*_, *y*_*ij*_)+*ς*(*x*_*ij*_, *y*_*ij*_) representing the weight between *x*_*ij*_ and *y*_*ij*_, and the output value is between [0, 1]. The larger the value, the higher the weight. Suppose that the chaotic set of the sports industry project *n* is ID and ID = {*a*_*i*_, *b*_*i*_, *d*_*i*_}, where *a*_*i*_ is chaotic (completely irregular = 1, rule = 2, and extraordinary rule = 0), *b*_*i*_ is the weight between industrial agglomeration and spatial governance (0 ∼ 0.3 = 1, 0.3∼0.6 = 2, and 0.6∼0.9 = 3), and *d*_*i*_ is the optimization situation (optimized = 1 and not optimized = 0), and the formula for the sports industry project optimization is expressed as follows:

(1) $$\begin{array}{c} N=\int_{0}^{\infty }\prod \left[\sum_{i,j}^{\infty }f\left(x_{ij},y_{ij}\right)+\varsigma \right]+\sum_{i}^{\infty }{\text{ID}}_{i}. \end{array}$$

Suppose that the governance mode of the sports industry project *n*_*i*_ is TR, TR = {*f*_*i*_, *g*_*i*_, *h*_*i*_}, *f*_*i*_ is spatial governance (regional spatial governance = 1 and overall spatial governance = 2), *g*_*i*_ is the governance mode (project integration = 1, project compression = 2 and project elimination = 3), *h*_*i*_ is policy, folk custom, infrastructure, and other uncertain factors, the formula is expressed as follows:

(2) $$\begin{array}{c} h_{i}=A_{i}\cdot f\left(x_{ij},y_{ij}\right), \end{array}$$

where ${\hat{x}}_{ij}$ is the projection of *x*_*ij*_ sports industry project aggregation, ${\hat{y}}_{ij}$ is the projection of*y*_*ij*_ spatial governance, and *A*_*i*_=*A*_*i*_=*∂ς*/(*∂x*_*ij*_ · *∂y*_*ij*_). The specific results are shown in Figure 4.

The article "Analysis and Research on Sustainable Development Factors of the Sports Industry Based on Chaos Theory" was published in 2022. Journal: J Environ Public Health.

It can be seen in Figure 4(a) that after projection processing, the interference attribute of the *z* axis in the original data will be removed, and the three-dimensional data will be changed into the two-dimensional data so as to reduce the impact of irrelevant attributes on sports industry agglomeration and spatial governance optimization.

### 3.4. Construction of the Optimization Algorithm under Chaos Theory

Zhou et al. proposed that the purpose of optimizing decision-making was to improve the rationality of the aggregation degree and spatial governance and reduce the amount of redundant data caused by sports policy and sports project development [15]. *K*-clustering can be used to process the aggregation degree and spatial governance data. The number of Fourier stages is centered on the preset threshold, the fluctuation of amplitude is carried out, and the relevant parameters and data are processed to make the final output result close to the threshold. At the same time, *K*-clustering can propose irrelevant data, extract eigenvalues that meet relevant requirements, and reduce the preprocessing capacity of data. The specific formula is expressed as follows.

(3) $$\begin{array}{c} \left|S\right|=\left\{\begin{array}{c} \sum_{i=0}^{n}x_{i},y_{i}\;x,y,\\ \sum_{i=0}^{n}e_{i}^{j\left(2\pi /2\right)\left(x_{i},y_{i}\right)}. \end{array}\right. \end{array}$$

Among them, *S* is the aggregation degree and the spatial governance number range of *K*-clustering. Since the information boundary *S* belongs to the fuzzy value, it can be identified by an approximate value.

The article "Analysis and Research on Sustainable Development Factors of the Sports Industry Based on Chaos Theory" was published in 2022. Journal: J Environ Public Health.

### 3.5. Weight Determination

Weight is not only the importance of evaluating various indicators in the sports industry but also the condition for industrial agglomeration and spatial governance optimization. It can make better decision-making analysis according to the objective situation. In the past, the weight of sports industry was calculated by a simple overall average and then analyzed layer by layer. However, the traditional method is suitable for a small amount of data calculation and not suitable for a large amount of data analysis. Therefore, the previous weight calculation methods cannot calculate the agglomeration and spatial governance of the sports industry. In this paper, the weight calculation method of the Lyapunov function is adopted, and the proportion of each parameter is calculated by the dichotomy of the weight sum and new weight. The specific calculation formula is expressed as follows:

(4) $$\begin{array}{c} w\left(x,y,G\right)=\left\{\begin{array}{c} \frac{H\cdot G_{ij}}{G_{i}+G_{j}},\\ w_{i}\left(x_{i},y_{i},G_{ij}\right)+\frac{1}{2}{\overset{⌢}{\varsigma }}_{i}\tau^{-1}. \end{array}\right. \end{array}$$

Among them, *G*_*i*_ is the frequency of *i* sports in the whole sports industry, *G*_*j*_ is the proportion of sports in dimension *j*, *H* is the coordination function between *G*_*i*_ and *G*_*j*_ (constant term), *w*_*i*_ is the proportion of *i* sports, $\overset{⌢}{\varsigma }$ is the projection of coordination function, *τ* is the average value of sports, and *τ* is a constant term (different values of different sports).

## 4. Result Output of Sports Industry Agglomeration and Spatial Governance Based on Chaos Theory

### 4.1. Constraints of Data Collection in the Sports Industry

In order to ensure that the optimization treatment results meet the requirements of chaos theory, the collected data shall be subject to the constraints of metropolis criteria to judge whether the data are effective. If the data are valid, the later calculation can be carried out; otherwise, the value will be eliminated. At the same time, metropolis accepted the criteria to assign values to sports industry data (structured = 1 and unstructured = 0), laying the foundation for later matrix construction and result output. In addition, metropolis acceptance criteria can make secondary judgment on the sports industry data that have been included and screened and eliminate noncharacteristic values. The specific calculation formula is expressed as follows:

(5) $$\begin{array}{c} F\left(x,y,\varsigma \right)\left\{\begin{array}{cc} T_{i}=T_{i+1}\neq 0, & \text{take in,}\\ T_{i}>or<T_{i+1}≃0 & \text{delte.} \end{array}\right. \end{array}$$

The sports industry items included in the calculation are taken as the initial value, and the iterative calculation is carried out to ensure that the sports industry with different dimensions *J* can be calculated accurately and play the irregular optimization role of chaos theory. In addition, the setting of constraints can also prevent local extremum from becoming an eigenvalue and improve the accuracy of governance decision-making.

The article "Analysis and Research on Sustainable Development Factors of the Sports Industry Based on Chaos Theory" was published in 2022. Journal: J Environ Public Health.

### 4.2. Sports Industry Agglomeration and Spatial Governance Results in Different Dimensions

The characteristics of the chaos theory are multidimensional, complex, and irregular, so its information is affected not only by the sports industry but also by the dimensions of the time, space, and policy.

Suppose that the calculation is divided into the same time dimension *P*_*u*_ and the same region dimension *P*_*v*_, and all fitting values are projected into the *xy* coordinate system to achieve the overall calculation of different dimension values and obtain the values of each value, as shown in Figure 4(b). Suppose that the aggregation and spatial governance of sports industry is *P*, the chaotic calculation formula of the sports industry in different dimensions is expressed as follows:

(6) $$\begin{array}{c} P\left\{\begin{array}{cc} \prod \left[\sum_{1,1}^{\infty }f\left(x_{11},y_{11}\right)+\varsigma \right]+\sum_{1}^{\infty }{\text{ID}}_{1}, & P_{u},P_{v}=P_{mg},\\ \frac{\kappa \left(P_{u}-P_{\min}\right)}{P_{mg}-P_{\min}}, & P_{c}<P_{mg},\\ \frac{\lambda \left(P_{v}-P_{\min}\right)}{P_{mg}-P_{\min}}, & P_{v}<P_{mg}. \end{array}\right. \end{array}$$

∏[∑_1,1_^*∞*^*f*(*x*_11_, *y*_11_)+*ς*]+∑_1_^*∞*^ID_1_ is the initial value after *K*-clustering treatment, and *P*_*u*_, *P*_*v*_=*P*_*mg*_. *P*_min_ is the minimum value in the same time dimension, *P*_*mg*_ is the minimum value in the same space dimension, *κ* is the coefficient between different dimensions, and *λ* is the chaotic coefficient. According to the above formula, the interdimension coefficient and the chaos coefficient are set between each dimension to ensure the significance of the final calculation result. In conclusion, the sports industry data are given initial values before calculation so that the initial values meet the requirements of the metropolis acceptance criteria and *K*-clustering, so as to improve the accuracy of governance.

The article "Analysis and Research on Sustainable Development Factors of the Sports Industry Based on Chaos Theory" was published in 2022. Journal: J Environ Public Health.

### 4.3. Aggregation Degree and Spatial Governance Results of the Sports Industry

The aggregation degree output of the sports industry is *R* (accurate output = 1 and error output = 0). It is difficult to manage the space. *L* (1 to 5 levels, compared with the average value of the sports industry, the higher the value, the higher the governance effect). After completing the analysis of the parameter weight and initial value, the appropriate function is used to calculate the accuracy of relevant optimization decisions so as to obtain accurate output results of sports industry agglomeration and spatial governance. The specific calculation formula is expressed as follows:

(7) $$\begin{array}{c} \left\{\begin{array}{cc} R=\min\int_{i,j}^{n}\left(w_{i}\left(x_{i},y_{i},G_{ij}\right)\max\prod \left[\sum_{i,j}^{\infty }f\left(x_{ij},y_{ij}\right)+\varsigma \right]\cup \right]\pm A_{i}\cdot f\left({\hat{x}}_{i},{\hat{y}}_{i}\right), & R\in \left[0,1\right],\\ L=\min\int_{i,j}^{n}\left(w_{i}\left(x_{i},y_{i},G_{ij}\right)\max\left[\prod \sum_{i,j}^{\infty }f\left(x_{ij},y_{ij}\right)\cup \frac{H\cdot G_{ij}}{G_{i}+G_{j}}\right],F\left(x,y,\varsigma \right)\right]\pm A_{i}\cdot f\left({\hat{x}}_{i},{\hat{y}}_{i}\right), & \sum_{i=0}^{n}e_{i}^{j\left(2\pi /2\right)\left(x_{i}^{0},y_{i}\right)}\propto 0. \end{array}\right. \end{array}$$

Among them, *w*_*i*_(*x*_*i*_, *y*_*i*_, *G*_*ij*_) is the output result of the sports industry agglomeration degree and ∏max[∑_*i*,*j*_^*∞*^*f*(*x*_*ij*_, *y*_*ij*_)+((*H* · *G*_*ij*_)/(*G*_*i*_+*G*_*j*_))] is the output result of sports industry spatial governance. Among them, comparing the spatial governance output with the average standard of spatial governance in the sports industry, the result is >0.5, indicating that the spatial governance effect is good.

### 4.4. Optimization Steps of Sports Industry Agglomeration and Spatial Governance Based on Chaos Theory

The models in Sections 3.1∼3.2 shall be analyzed step by step and iteratively, and finally, the decision results of sports industry agglomeration and spatial governance shall be obtained. The specific steps are as follows:

1. Set the data nodes *N*,*N* = {*n*_1_*,n*_2_*...n*_*i*_}, and *n*_*i*_=∑_*i*,*j*_^*∞*^*f*(*x*_*ij*_, *y*_*ij*_)+*ς*(*x*_*ij*_, *y*_*ij*_). Conduct *K*-clustering processing on the collected data, judge metropolis acceptance criteria, calculate relevant results, and go to step 2.
2. Iterate the processed sports industry data, eliminate *P*_*u*_ and *P*_*v*_ attributes, calculate the aggregation degree, and output them as *R* and *L.* After the analysis of the parameter weight and initial value, the appropriate function is used to calculate the accuracy of relevant optimization decisions.
3. Each time, the results of iterative calculation shall be judged and compared with Max (*R,L*). If the result is greater than Max (*R, L*), it meets the requirements and is included in the *R* and *L* sets, otherwise it is eliminated. At the same time, record the calculation time *t* of each result to judge whether the time is >0. If the obtained time is >0, it indicates that the treatment result meets the requirements of time series in the chaos theory, otherwise the data are eliminated.
4. Judge whether all the sports industry project nodes *i* are calculated. If all the projects are traversed, the calculation is terminated; otherwise, repeat step 2 until the relevant requirements are met.
5. Finally, the Max (*R,L*) value is output, the governance calculation is completed, and the calculation results are output.

The article "Analysis and Research on Sustainable Development Factors of the Sports Industry Based on Chaos Theory" was published in 2022. Journal: J Environ Public Health.

The results are shown in Figure 5.

## 5. The Case Analysis of Sports Industry Agglomeration and Spatial Governance Optimization

### 5.1. The Data Sources

In order to ensure the accuracy and effectiveness of the data, the random method is used for data extraction and the chaotic theory algorithm is compared with the previous genetic algorithm. A total of 7 provincial regions, 9 municipal regions, 9 sports events, and 6 related industries were investigated. The results are shown in Figure 6.

In order to verify the validity of the aforementioned data, it is necessary to analyze the validity and reliability of the data collected in Figure 7 to judge whether the relevant data meet the expected requirements. The results are shown in Figure 7.

It can be seen from Figure 7 that the collected sports industry data have good credibility and validity, and all values are positive. The provincial credit rating is concentrated at 1.5, the municipal credit rating is concentrated at 6.5, sports events are concentrated at 4.5, and related industries are concentrated at 1.9. It can be seen that the sports industry data collected in this paper are relatively concentrated, and there is no large dispersion, which can be used as the basis for later data analysis. In addition, the random sampling method is adopted in this paper, and the data obtained are highly representative, which show that the sampling sample meets the requirements of chaos theory analysis. The above results are consistent with the research conducted by Zhou et al. [15].

The article "Analysis and Research on Sustainable Development Factors of the Sports Industry Based on Chaos Theory" was published in 2022. Journal: J Environ Public Health.

### 5.2. Calculation of the Sports Industry Agglomeration Degree

For the survey data, the optimization decision-making method of the chaos theory and the previous genetic algorithm are used to analyze the sports industry aggregation degree of the two algorithms. The analysis results are shown in Figure 8.

According to the analysis of the aggregation degree illustrated in Figure 8, the aggregation degree of the sports industry based on the chaos theory is higher than that of previous genetic algorithms. On the basis of the same sports events and the chaos theory, the aggregation degree of sports industry is greater than 95% and the average aggregation degree is 95.82 ± 2.3, while the aggregation degree of the genetic algorithm is greater than 90% and the average aggregation degree is 92.82 ± 1.3. There is a significant difference between them (*X*^2^ = 2.32, *P* < 0.05). The reason for the above differences is that the chaos theory eliminates the *P*_*u*_ and *P*_*v*_ attributes in the sports industry, making the recording degree of the sports industry data better. In addition, the irregular and nonqualitative analysis method of the chaos theory can realize the analysis of multidimensional sports industry data, extract the key information value, reduce the redundant data useless to the concentration degree of the sports industry, and realize the massive analysis of the sports industry data. Compared with the genetic algorithm, the chaos theory has two advantages. On the one hand, the chaos theory does not need to sort out the sports industry data but only needs to extract the key values to realize the data analysis. On the other hand, the nonqualitative analysis method of the chaos theory can analyze the data relevance in the sports industry and eliminate the repetitive data and attributes. The above results are consistent with the research conducted by Chen et al. [16].

### 5.3. Space Governance Calculation of the Sports Industry

The analysis method in Section 4.2 is still used to calculate the spatial governance of the sports industry. The calculation results are shown in Figure 9.

Through the spatial governance analysis demonstrated in Figure 9, it can be seen that the spatial governance algorithm of the sports industry based on the chaos theory is more effective and it has been concentrated in the region at 867 times, while the genetic algorithm needs to be concentrated at 2340. In addition, the spatial governance algorithm of the sports industry based on the chaos theory changes only 0.04%, which is significantly higher than 0.1% of the genetic algorithm. The reason for the above differences is that due to the irregular analysis of the chaos theory, there are more records of spatial governance data of the sports industry in the early stage and a large number of data screening in the later stage. In addition, the irregular and nonqualitative analysis method of the chaos theory can realize multidimensional spatial compression and reduce the useless redundant data in the sports industry space, such as policy, region, and custom. The above results are consistent with the research conducted by Kundrák et al. [17]. Compared with the genetic algorithm, the improved chaos theory proposed in this paper has better advantages in space compression and simplified analysis. In addition, the irregular and non-qualitative analysis method of the chaos theory can realize multidimensional spatial compression and reduce the useless redundant data in the sports industry space, such as policy, region, and custom. Compared with the genetic algorithm, the chaos theory is better in space compression and reduction to analysis. It can be seen from the analysis in Figure 9 that the reduced dimension analysis of chaos theory and irregular data analysis can effectively reduce the volatility factors in the data. At the same time during irregular analysis, the amount of data and complexity are preprocessed to enhance the effect of spatial governance. The chaos theory uses multidimensional projection to simplify the complex sports spatial data, which can increase the number of spatial data processing, reduce the complexity of spatial data, and realize the optimal analysis of sports spatial data. The above results are consistent with the research conducted by Li et al. [18].

The article "Analysis and Research on Sustainable Development Factors of the Sports Industry Based on Chaos Theory" was published in 2022. Journal: J Environ Public Health.

To sum up, the improved chaos theory model is superior to the genetic algorithm in terms of data reliability, spatial governance, data fusion, and fluctuation range of the sports industry and the incidence of the “local extreme value” is lower than that of the genetic algorithm, which has obvious overall advantages.

## 6. Conclusion

How to effectively use the infrastructure of the sports industry, improve the agglomeration of the sports industry, and rationally carry out the spatial distribution of the sports industry are problems to be solved urgently, which are also an important analysis goal for economic development. Based on the above background, this paper constructs an optimal decision-making model for the sports industry and economic development. Through the analysis of irregular data and nonlinear data in the sports industry, the model realizes the agglomeration of the sports industry and its own users of the space. First, the difficulties and starting points of the sports industry agglomeration are analyzed. It analyzes the redundant data and irregular data in the industry, and it is believed that finding out the key values in the sports industry data and eliminating the attribute values in the data are the key goals of optimization. Secondly, this paper selects two aspects of sports industry agglomeration and spatial governance and four parameters to analyze the weights and correlations between values. Through the correlation and weight, this paper constructs an optimal decision-making model for sports industry agglomeration and spatial governance based on the chaos theory, which provides an important reference for economic development. According to the chaos theory, the aggregation degree of the sports industry is greater than 95% and the variation range of spatial governance and the number of optimal results are obviously better than those of the genetic algorithm. Therefore, the optimization model based on the chaos theory can provide decision support for the sports industry. This paper does not analyze the prediction of industrial agglomeration and spatial governance, which will be analyzed in future research.

The article "Analysis and Research on Sustainable Development Factors of the Sports Industry Based on Chaos Theory" was published in 2022. Journal: J Environ Public Health.

Chaos theory is seldom used in sports research in the previous research results [19–23]. The optimization model based on the chaos theory can provide decision support for the sports industry. This paper does not analyze the prediction of industrial agglomeration and spatial governance, which will be analyzed in future research. The nature of the world is chaotic, and the sports industry system is also a complex and nonlinear chaotic system. The chaotic nature of the sports industry requires us to break through the traditional thinking paradigm of sports industry design and pursue new and dynamic design. The research mode of the sports industry exists under the guidance of nonlinear chaos theory. In reality, chaos and the traditional sports industry design mode exist in contradiction and there are differences between them. We should examine these contradictions and differences scientifically. Chaos theory is valuable and can be used for reference, which provides a new perspective for the development of the sports industry.

## Figures and Tables

**Figure 1:** Data collection of sports industry agglomeration and spatial governance based on chaos theory.

**Figure 2:** Sports industry agglomeration process.

**Figure 3:** Spatial governance scheme of the sports industry.

**Figure 4:** Sports industry data projection.

**Figure 5:** Optimization steps of sports industry agglomeration and spatial governance.

**Figure 6:** The sources of the survey data.

**Figure 7:** Reliability and validity results of the survey data.

**Figure 8:** Degree of sports industry agglomeration.

The article "Analysis and Research on Sustainable Development Factors of the Sports Industry Based on Chaos Theory" was published in 2022. Journal: J Environ Public Health.

**Figure 9:** Spatial governance of the sports industry.

**Table 1:** Core indicators of sports industry agglomeration and spatial governance.

Index category		Quantity	Quantity
Industrial agglomeration	Intraindustry agglomeration	16	Quantity
	Industrial agglomeration	18	Clothing, catering, and other related industries

Space governance	Regional space governance	10	Regional characteristics, regional scope, and governance
	Overall spatial distribution governance	12	Provincial governance and national governance

Data source: data released by the government and questionnaire.

## Data Availability

The data used to support the ﬁndings of this study are available from the corresponding author upon request.
